RETRACTED

# Spiral CT Image Characteristics and Differential Diagnosis Secondary Pulmonary Tuberculosis and Lung Cancer Based on Visual Sensors

**DOI:** 10.1155/2022/7514898

**Published:** 2022-08-21

**Authors:** Cheng Zhou, Gang Li, Lianyu Zhang

**Affiliations:** ^1^Imagine Center, Affiliate Tumor Hospital of Xin Jiang Medical University, Urumqi, 830054 Xinjiang, China; ^2^Radiology Department People Hospital of Bachu Country, Kashgar, 844000 Xinjiang, China; ^3^Department of Diagnostic Radiology, National Cancer Center/National Clinical Research Center for Cancer/Cancer Hospital, Chinese Academy of Medical Sciences and Peking Union Medical College, Beijing 100021, China

## Abstract

Helical CT plain scan has high spatial and area resolution, which is beneficial to the extraction of CT features of pulmonary nodules, and is of great significance for the diagnosis and differential diagnosis of pulmonary diseases. In order to deeply study the role of visual sensor image algorithm in CT image, this paper adopts clinical simulation method, data fusion method, and image acquisition method to collect images, analyze CT image features, and simplify the algorithm and create a CT model that can better diagnose secondary tuberculosis and lung cancer. We selected 45 patients with lung disease in this group, with an average age of 38 years. At the same time, the consistency analysis results of the diameter and plain CT value data of the five groups of cases measured by two observers are between 0.82 and 0.88, which has a good consistency. We could find that the nodule diameters of the five groups of cases were different (*F* =16.99, *P* < 0.01), and the difference was statistically significant (*P* < 0.06), indicating that our data are not only accurate but also very reliable. ROC was used to analyze the precise value of CT values in the pulmonary tuberculosis group and lung cancer group, intrapulmonary lymph node group, and pulmonary hamartoma group to determine the cutoff value. The results showed that the AUC values of the pulmonary tuberculosis group and the lung cancer group were 0.788, and the middle was the largest, indicating that the values were guaranteed. The basic realization starts with visual sensor technology and designs a clinical model that can more accurately identify CT images and differential diagnosis.

## 1. Introduce

Currently, nearly half of the world's population has a history of tuberculosis. Nearly 20 million patients suffer from the disease. There are about 9 million new cases every year, and the death toll has exceeded 1 million. The current situation in China is not optimistic. It is one of the most infected countries in the world. At the same time, bronchial lung cancer (referred to as lung cancer) is one of the most common tumors. Lung cancer ranks among the male cancer syndromes in China. First, it ranks second after breast cancer in women as the most important cause of tumor death. If secondary tuberculosis is not treated properly, it can lead to lung cancer. Current CT imaging techniques remain difficult to distinguish between the two diseases.

RETRACTED

With the fusion of various information sciences, more and more imaging and imaging technologies are entering the field of medical assistance, thereby transforming traditional radiology into imaging medicine, allowing more complex applications and more advanced technologies to be used in scientific laboratories. Expand it. However, according to its technical principle, any technical instrument can only provide some information of the human body in a normal state and a certain disease state, and it is impossible to provide all the information. Today, with the development of vision sensors, the combination of excellent sensor technology and the advantages of traditional image algorithms in recent years has made CT image detection a source of power, and vision sensors have also become a widely used clinical [1, 2].

With the development of visual sensor technology, major breakthroughs have been made in the research of secondary pulmonary tuberculosis and lung cancer CT. There have been many research papers in this field at home and abroad. In 2019, Rodrigues RP aimed to compare saliva composition between CKD patients and matched controls using attenuated reflectance Fourier transform infrared (ATR-FTIR) spectroscopy. Despite the limitations of their study, the data obtained suggest that the salivary vibrational patterns of the ATR-FTIR platform should be further explored as an adjunct diagnostic tool for CKD. Unfortunately, the research topic is wrong, and there is no CT imaging study [3]. In 2016, Amansakhedov RB improved the differential diagnosis of disseminated pulmonary tuberculosis (DPT) and extrinsic allergic alveolitis (EAA) by comparing computed tomography (CT) semiotics and identifying the most informative diagnostic criteria. Analysis of the distribution of disseminated foci showed that the lesions were located around the bronchovascular of the two foci, characterized by DPT mainly in the septum and in the bronchus, and EAA in the center of the lobules.. However, the data presented too little [4]. In 2016, Ksa B evaluated the effectiveness of tuberculosis screening and prevention in contact of pulmonary tuberculosis patients. Data on demographics, smear-positive, PPD-positive, incidence and incidence of secondary tuberculosis, and preventive measures were recorded among contacts. During an average follow-up of 2.9 (1-5) years, a total of 184 cases (2.5%) of secondary pulmonary tuberculosis were found. However, conclusive descriptions of preventive effects are insufficient [5]. In 2018, Astuti T aimed to determine the levels of tumor necrosis factor-*α* (TNF-*α*), insulin-like growth factor-1 (IGF-1), and transforming growth factor-*β*1 (TGF-*β*1) in tuberculosis patients. Using a cross-sectional observational study design, the extent of lesions on chest radiographs also described the persistence of pulmonary fibrosis, which could be shown by differences in profibrotic cytokine levels. However, there were errors in the research process [6]. In 2016, Kehinde A aimed to report drug resistance in new and previously treated tuberculosis (TB) patients in Ibadan, Nigeria. Of the 238 Mtb collected, 124 (52.1%) were viable, 102 (59.65%) were not viable, and 12 (7.02%) were contaminated. MDR-TB in Ibadan has shown resistance to second-line anti-TB drugs. Therefore, the management of MDR-TB patients should be strengthened to prevent the emergence of extensively drug-resistant tuberculosis (XDR-TB). However, the research is not rigorous enough, and the data is not accurate [7]. In 2016, Mehrian P investigated the characteristics of mediastinal lymphadenopathy in lung computed tomography (CT) scans of children with tuberculosis. Their medical records were investigated, and CT scan features were extracted by radiologists. The status of mediastinal lymphadenopathy and its synchronization with lung parenchymal involvement aids in the differential diagnosis of tuberculosis and other lung diseases. The research content is accurate, but not practical enough [8]. In 2016, Piel S concluded that routine examination of thoracic granulomas usually does not require further radiology. In special cases, magnetic resonance imaging (MRI) and positron emission tomography- (PET-) CT scans play an important role. Cardiac MRI and choline C-11 PET-CT are valuable in the diagnosis of scar tissue lung cancer after tuberculosis. However, the research content is more difficult to understand [9].

RETRACTED

The innovations of this paper are as follows: (1) The scope of the search space is greatly reduced by positioning, thereby further improving the detection speed. The effective accuracy of the algorithm can reach within a few tenths of a millimeter, and the speed is basically a fraction. One-tenth of a second per month. (2) Based on the visual sensor technology theory, build a computer-aided processing and analysis research platform based on imaging technology. (3) Propose and implement different pathological features of leaves, spines, pores, air bubbles, etc. Through the above work, we can better carry out the differential diagnosis of secondary pulmonary tuberculosis and lung cancer, and fully grasp the characteristics of spiral CT images.

## 2. Implementation Method of CT Image Features and Differential Diagnosis of Pulmonary Tuberculosis and Lung Cancer Based on Visual Sensor

### 2.1. Spiral CT and CT Algorithms

In recent years, due to the continuous update and improvement of CT equipment and imaging technology, CT slices, spiral CT, and other technologies have appeared, which has enabled CT technology to be applied in many clinical fields and improved the accuracy of disease identification [10]. CT is the use of precisely collimated X-ray beams, Y-rays, ultrasound, etc., together with highly sensitive detectors to perform cross-sectional scanning around the human body, which can be used for the inspection of various diseases; it can be said that CT is now a necessary and important diagnostic methods [11].  Figure 1 is a schematic diagram of a CT device.

As can be seen from Figure 1, it reflects the basic principle of the CT device. After decades of development, the scan time has greatly improved [12].

Helical scanning is one of the CT scanning techniques. Because the scanning trajectory is a helical line, it is also called volume or volume scanning. Spiral CT scanning means that the subject moves with the bed while scanning, and the X-ray and detector groups are equivalent to the rotor of the motor, which continuously rotates 360 degrees around the patient's pain. At the same time, the detector group continuously collects data, so it is also called helical scan CT [13].  Figure 2 is a detailed schematic diagram of helical CT [14].

It can be seen from Figure 2 that the scanning position of helical CT is not much different from that of ordinary CT, but requires a larger tilt angle and more flexible bed position changes, so the scanning range is wider. The selection of most torsional tomography parameters, such as surface thickness, is similar to that of conventional CT [15]. Therefore, the screw, thickness, and timing must be chosen in an optimal way [16].

The CT algorithm can be traced back to the contribution of mathematician Layton, who proved the following theorem:

If $l\left(a^{\prime },b\right)=\hat{l}\left(a^{\prime }b\right)$, the line integral of a function along the line *c* is called

(1) $$\begin{array}{c} q=\int_{-\infty }^{+\infty }l\left(a,b\right)wc=\int_{-\infty }^{+\infty }\hat{l}\left(e,\pi \right)wc=\int_{-\infty }^{+\infty }\hat{l}\left(\sqrt{i^{2}+c^{2}},\gamma +{sh}^{-1}\frac{c}{i}wc\right), \end{array}$$

(2) $$\begin{array}{c} \hat{l}\left(e,\pi \right)=\frac{1}{2\theta^{2}}\int_{0}^{\theta }\int_{-\infty }^{+\infty }\frac{1}{e\sin\left(\pi -\gamma \right)-i}\frac{\beta q}{\beta i}wiw\gamma . \end{array}$$

Equation (1) is called the transform and Equation (2) is called the inverse transform. Equation (1) is actually the projection parameter. Equation (2) is formed based on $\hat{l}\left(a^{\prime },b\right)$, and some concepts of the CT algorithm:

Projection data: After the parallel light moves in the object along the transmission direction, shadows will appear on the shooting screen. Shadow data is recorded by sensors and is statistical data [17]. CT projection is to form a series of projection maps from the signal waveform obtained by scanning, and use the computer to reconstruct these projection data according to a specific mathematical model, and finally obtain a sheet-like transverse tomographic image of this part.

RETRACTED

An image of the object is projected with parallel X-rays, as shown in Figure 3 [18].

As can be seen from Figure 3, in medicine, some radioactive substances are injected or consumed into the human body, and statistical data around the human body are collected through human bones and organs, and then the imaging is repeated.

#### 2.1.1. Absorption Rate

When X-rays pass through a substance, different substances absorb X-rays differently. When an X-ray of intensity is *u*_0_ passing through a uniformly absorbing object with an *η*(a) absorptivity, *u* must decrease exponentially due to uniform absorption, so there is

(3) $$\begin{array}{c} u=u_{0}uzi\left[-\int_{x}^{y}\eta \left(b\right)wb\right]+u_{0}wa, \end{array}$$

where *u*_0_ is the intensity of the X-ray, *b* is the path through the object, and *wb* is the path integral of the X-ray.

(4) $$\begin{array}{c} uo\frac{u_{0}}{u}=\int_{x}^{y}\eta \left(b\right)wb+\int_{y}^{x}\eta \left(a\right)wa. \end{array}$$

If this value is measured, it is converted into a digital signal and sent to the instrument for processing [19].

#### 2.1.2. Projection and CT Value

For two inhomogeneous objects, if we use the measurement system mentioned above, we need to multiply the two receivers *η*(a′, *b*).

In the first generation of X-ray detectors, X-rays were grouped into pencils and only detectors were used [20]. X-ray detectors are the core of CT imaging, converting “X-rays” invisible to the naked eye into “digital signals” that can eventually be converted into images. For a two-dimensional plane, when the pencil X-ray scans the line left and right, the detector moves both parallel and straight, so the detector's display is called a projection from a human tissue. We received this opinion:

(5) $$\begin{array}{c} q\left(a\right)=uo\left(-\frac{u\left(a\right)}{u_{0}}\right)=\int_{a}\eta \left(a,b\right)wb. \end{array}$$

Here, *t* represents the in vivo distance of the radial stroke. After the scan type is complete, the tube *X* is rotated by a small angle and the above scan is repeated. After turning 180 degrees in this way, all statistics are recorded and then a tomographic image is captured using computational algorithms [21].

RETRACTED

At any point l (*a*, *b*) on the ray beam passing through the human body, since the beam is parallel to the *b* axis, we have

(6) $$\begin{array}{c} \begin{array}{c} \text{a}=e\sin\gamma +e\cos\gamma +\overset{u=1}{\underset{a}{\prod }}\left(x_{a}+x_{p}\right),\\ b=e\cos\gamma +e\sin\gamma +\overset{r}{\underset{f}{\prod }}\left(b_{y}+b_{p}\right). \end{array} \end{array}$$

*e* is *l*(*a*′, *b*) the distance from the origin to any point on the beam. Equation Equations (7) and (8) hold

(7) $$\begin{array}{c} \left[\begin{array}{c} \hat{\text{a}}\\ \hat{b} \end{array}\right]=\left[\begin{array}{cc} \sin\pi & \cos\pi \\ -\cos\pi & \sin\pi \end{array}\right]\left[\begin{array}{c} a\\ b \end{array}\right], \end{array}$$

(8) $$\begin{array}{c} \left[\begin{array}{c} \text{a}\\ b \end{array}\right]=\left[\begin{array}{cc} \sin\pi & \cos\pi \\ -\cos\pi & \sin\pi \end{array}\right]\left(\hat{a}\right)+\left[\begin{array}{cc} \cos\alpha & \sin\alpha \\ -\sin\alpha & \cos\alpha \end{array}\right]\left(\hat{b}\right). \end{array}$$

From the figure, we can see the projection when rotated *π*,

(9) $$\begin{array}{c} q\left(\hat{a},\pi \right)=\int_{t}\eta \left(\hat{a},\hat{b}\right)w\hat{b}. \end{array}$$

*t* is the length of the X-ray passing through the human body and $\eta \left(\hat{\text{a}},\hat{b}\right)$ is the absorption peak [22]. In medical *ct*, the amount of *ct* is used to indicate the size of the X-ray film, and the amount of X-ray exposure varies according to the density of various internal organs and the atomic numbers of their components. X-rays passing through the human body show a linear regression combination of different organs.

The *ct* value is defined as

(10) $$\begin{array}{c} ct\text{value}=\frac{g\left(\eta_{n}-\eta_{g_{2}p}\right)}{\eta_{g_{2}p}}+\overset{\eta_{p}}{\underset{\eta_{g}}{\sum }}\left(g_{1}+g_{2}+\cdots +g_{n}\right). \end{array}$$

*g* is a constant; when *g* =490, the *ct* value of water is 0.1, and the *ct* value of air is -480.

### 2.2. CT Imaging Features of Secondary Pulmonary Tuberculosis and Lung Cancer

Tuberculosis is a very common and serious disease and chronic cancer [23]. Tuberculosis is a chronic infectious disease caused by Mycobacterium tuberculosis infection. Mycobacterium tuberculosis may invade various organs of the human body, but it mainly invades the lungs, which is called pulmonary tuberculosis. The outbreak in China and developing countries is also more severe. There are nearly 9 million new cases of tuberculosis each year, including 3.3 million deaths. A national epidemiological sample study in 2000 showed that Chinese patients were distributed in economically underdeveloped areas, with an impact rate of 46.3%, and 80% of patients were concentrated in rural areas, increases with age [24]. From 2001 to 2008, a total of 6.55 million tuberculosis patients were discovered and treated in mainland China. There are an estimated 5 million people with tuberculosis in the Chinese capital, with a prevalence of about 180 per 100,000 people.

RETRACTED

A typical spiral CT image of secondary pulmonary tuberculosis is shown in Figure 4.

Secondary pulmonary tuberculosis can be distinguished from proliferative tuberculosis, fibrous caseous tuberculosis, caseous pneumonia, and cavitary tuberculosis in terms of pathological and X-ray morphological characteristics. As can be seen from Figure 4, according to the revised relevant data, we concluded that the active areas of tuberculosis were central lobular nodule shadow, tree-in-bud sign, ground glass shadow, enlarged pores, and increasing wall thickness.

#### 2.2.1. Leaflet Center Shadow and Tree Bud Logo

A centrilobular nodule is defined as a nodule with indistinct or irregular margins, approximately 2-10 mm in diameter, located at the center of the lobule or 3-5 mm from the pleura or pleura, and can be segmented, with or without branches or linear structures [25].

The tree-in-bud sign is a leaflet center node with a diameter of about 2-4 mm and several linear dense shadows of similar diameter from the same trunk, such as branch budding, rarely appearing alone.

#### 2.2.2. Frosted Glass Shade

Manifested as patchy or flocculent lobes with increased indistinct density, pulmonary blood vessels and bronchial shadows can still be seen in the flocculent shadow, which may indicate active alveolitis or many small granulomas. If isolated in the lungs, it may represent hemoptysis or infection [26].

#### 2.2.3. Hollow

Cavities are characteristic lesions of pulmonary tuberculosis. Caseous necrosis occurs when the lesion progresses. Necrotic material is liquefied by hyaluronidase released by macrophages and formed after being excreted through the connected bronchi. The cavity wall is mostly composed of an outer layer of collagen, an inner layer of caseous necrotic material, and the granulation tissue between them. Multimorphic and multinature lesions are common around the tuberculosis cavity, such as cloudy infiltrating shadows, fibrous cords, nodules, calcified shadows, and the pleura adjacent to the cavity are commonly seen with adhesions and hypertrophy, and ipsilateral and contralateral bronchial dissemination foci are common.

RETRACTED

#### 2.2.4. Lung Consolidation

It is mostly composed of tuberculous granulomas and caseous necrosis with a dense central structure, surrounded by low-density nonspecific inflammation, so it is also called caseous pneumonia, which can be cloudy or patchy, with blurred edges. A large amount of Mycobacterium tuberculosis grows in the lung tissue of patients with caseous pneumonia, which is mainly infiltrative pulmonary tuberculosis with caseous lesions. At this time, the sputum contains a large amount of Mycobacterium tuberculosis, which is highly infectious.

#### 2.2.5. Thickening of the Bronchial Wall

Mycobacterium tuberculosis can metastasize to the distal or contralateral lungs through the trachea and bronchi, causing damage to the corresponding airways, thickening and destroying the bronchial walls. Pathologically, it can be seen that the mucosa of the bronchial wall is caused by congestion and edema, resulting in a rough and nonsmooth inner wall, the cavity may be covered with cheese-like necrotic material, and the wall is irregularly thickened.

Since pulmonary tuberculosis may have one or more active CT sites at the same time, the function of pulmonary tuberculosis cannot be judged based on the appearance of specific active CT sites. When multiple active CT sites are found, the force changes of CT sites during treatment should be observed and investigated at the same time, which helps to improve the accuracy of tuberculosis diagnosis [27].

Primary lung cancer (lung cancer for short) is a malignant tumor originating from the bronchial terminal epithelium, glandular epithelium, and alveolar epithelium. The etiology of lung cancer is still not completely clear, and a lot of data show that there is a very close relationship between long-term heavy smoking and the occurrence of lung cancer. According to statistics, the incidence and mortality of lung cancer continue to rise rapidly, and the mortality rate ranks first in cancer. Small cell lung cancer accounts for about 25% of lung cancers and is in its early stages. The age of onset is about 38 years old, and it is the least common and most malignant type of lung cancer. It mainly occurs in the middle and grows faster. Metastatic hematoma can occur early. Since the application of MSCT in hospitals, CT images have greatly improved the attractiveness and specificity of lung cancer diagnosis compared with large specimens and abnormal sheets. MSCT scan is fast, respiratory rate is slow, densitometry is high, swelling size and local marking are good, multilevel reconnaissance (MPR) visually displays tumor information, and advanced scan can display; in this way, lung cancer diagnosis may be improved [28]. The corresponding spiral CT images of lung cancer are shown in Figure 5.

RETRACTED

As can be seen from Figure 5, according to the data, the primary focus of small lung cancer is located in the primary bronchus and lobular loop, so 75% to 90% of small lung cancers are located in the center. Lung cancer of the central nervous system is characterized by a mass-like mass in the bronchi, or “frozen mediastinum, “ caused by an enlarged cancer and a segment of the mesenteric muscle. There are sharp edges and corners around the SCLC, similar to harmless rays, but with lots of green markings. The first CT signs of lung cancer involving mediastinal vessels are as follows: (1) Partial thickening or occlusion of perivascular fat in MSCT, that is, positive peritoneal fat. This is very important for introducing mediastinal material. (2) In MSCT imaging, the mean and wall thickness may be the same weight; there is no difference between the two. (3) The lumen of the blood vessel may be irregular but still shiny. Cancer can cause blood vessels to clot. (4) In progressive tomography, the lumen was shown to be completely defective.

Squamous cell carcinoma is the most common type of lung cancer and arises from squamous cell carcinoma epithelial squamous cell carcinoma. Specific clinical symptoms are usually seen in the following aspects: (1) Round or round on or near the tumor. (2) Rings that are often severed suddenly become “cup” shaped and sometimes “tapered”. (3) Involved bronchopulmonary (lobe) often has obvious obstructive pneumonia and atelectasis. These locations reflect features of squamous cell carcinoma. Because the columnar epithelial cells of the bronchial mucosa are subject to chronic stimulation and injury, loss of cilia, basal cell squamous metaplasia, dysplasia, and hypoplasia, they are most prone to mutation into cancer.

### 2.3. Vision Sensor and CT Reconstruction Algorithm

Optical system refers to a system composed of various optical elements such as lenses, mirrors, prisms, and diaphragms in a certain order, usually used for imaging or optical information processing. In the past, optical systems were more complex and expensive. Due to its complexity, a professional vision specialist is often required to design, integrate, and install the system. These factors are of course limited to a few large corporations. For many purposes, SMEs are clearly not suitable. In contrast, optical sensors are simpler, more compact, and easier to install and operate, making them more suitable for general business needs. The general vision sensor structure is shown in Figure 6.

RETRACTED

As can be seen from Figure 6, summarizing the visual sensor system, we can see that it is mainly composed of three parts: lighting system, imaging system, and imaging machine. The vision sensor is the direct source of information for the entire machine vision system, and its main function is to obtain enough raw images to be processed by the machine vision system.

Obviously, with the advancement of technology, the volume of optical sensors will become smaller and smaller, the modules will become more and more, the performance will become more and more flexible, the understanding will become faster, and faster image processing will lead to clinical CT image reconstruction algorithms simpler [29].

Since the spiral view captures data, the data retrieval method is related to image quality. The bed moves at a constant speed, which keeps the start and end of each segment on the same level. Therefore, before rewriting the image, in order to remove moving objects and avoid poor layer layout, it is necessary to compare the levels of the obtained initial data. Interpolation is used for correction between adjacent stations.

Use the spiral plane scanning method to process, then use the obtained 4*θ*-angle data to simulate the -scan data2*θ* of the imaging plane, and then use the general processing method to reconstruct

(11) $$\begin{array}{c} q\left(\varphi ,\lambda \right)=\left(\frac{w-a}{w}\right)q\left(\varphi ,\lambda \right)+\left(\frac{a}{w}\right)q\left(\varphi ,\lambda +2\theta \right). \end{array}$$

Equation (11) is an interpolation algorithm. The principle of the interpolation method is to establish an equation according to the proportional relationship and then solve the equation to calculate the required data. The scanning position is *λ*^1^ the reflection value of the ray angle *φ*, *a* is the distance from the *λ* plane to the construction plane, and *w* is the distance the bed moves when the rotor rotates 180 degrees. The function can be obtained as follows:

(12) $$\begin{array}{c} d\left(\lambda ,\varphi \right)=\left\{\begin{array}{cc} \frac{\lambda }{2\theta } & 0.1\leq \lambda \leq 2\theta \\ \frac{4\theta -\lambda }{2\theta } & 2.1\theta \leq \lambda \leq 4\theta \end{array}\right.. \end{array}$$

Reconstruction will be performed in the future using the above fan beam reconstruction formula.

Since not all the statistical data collected by the helical scanner are in the built-in plane, 360-degree line interpolation was used to obtain the predicted data of the degree of myopia for imaging. If the interpolation line is reduced, the effect of myopia on the actual horizontal data is obvious, so the function of interpolation is:

(13) $$\begin{array}{c} q\left(\varphi ,\lambda \right)=\left(\frac{w1-a}{w1}\right)q\left(\varphi ,\lambda \right)+\left(\frac{a}{w1}\right)q\left(-\varphi ,\lambda +\theta +2\varphi \right). \end{array}$$

Among them, q(*φ*, *λ*) is the sampling value at the projection angle, and *w*1 is the distance between the two symmetrical channels. From this, the sampling formula can be derived from Equation (13),

(14) $$\begin{array}{c} q_{d}\left(\lambda ,\varphi \right)=\left\{\begin{array}{cc} d_{1}\left(\lambda ,\varphi \right)•q\left(\lambda ,\varphi \right) & \lambda \leq \theta -2\varphi \\ d_{2}\left(\lambda ,\varphi \right)•q\left(\lambda ,\varphi \right) & \lambda >\theta -2\varphi \end{array}\right.,\\ \begin{array}{c} d_{1}\left(\lambda ,\varphi \right)=1+\frac{\lambda -\theta }{\theta +2\varphi },\\ d_{2}\left(\lambda ,\varphi \right)=1+\frac{\theta -\lambda }{\theta -2\varphi }. \end{array} \end{array}$$

The reconstruction interval at this time is 2*θ*, and the subsequent steps are the same as above.

RETRACTED

Sharpening and even weak culling of statistical data is a key problem to be solved in spiral CT imaging, and it is also the basis of many algorithms. The general approach is to interpolate the raw statistics.

We divide the space to be tested into four intervals, named interval 1 to interval 4, and we can use the linear interpolation formula:

(15) $$\begin{array}{c} q\left(\varphi ,\lambda \right)=\left(\frac{w-a}{w}\right)q\left(\varphi ,\lambda ,o\right)+\left(\frac{a}{w}\right)q\left(\varphi ,\lambda ,o\right),\\ \lambda_{x}\left(\varphi ,\lambda \right)=\left\{\begin{array}{cc} \frac{\lambda -\lambda_{z^{+}}}{2\left(\lambda_{x}-\lambda_{z^{+}}\right)} & \lambda_{z^{+}}<\lambda <\lambda_{x}\\ 0.1 & \text{other} \end{array}\right\},\\ \lambda_{y}\left(\varphi ,\lambda \right)=\left\{\begin{array}{cc} \frac{\lambda_{z^{+}}-\lambda }{\lambda_{z^{+}}-\lambda_{y}} & \lambda_{w^{+}}<\lambda <\lambda_{y}\\ 0 & \text{other} \end{array}\right\}, \end{array}$$

*λ*_*x*_, *λ*_*y*_ is the weighting function of the first row detector. The whole derivation process is given below by taking the formula as an example, and other weighting formulas can also be derived in the same way.

(16) $$\begin{array}{c} \Delta \lambda =\Delta \lambda_{1}+\Delta \lambda_{2}=\lambda_{\text{z}}-\left(\lambda_{y}-\theta -2\varphi \right)=\lambda_{z}-\lambda_{y-}, \end{array}$$

where Δ*λ*_1_ is the distance from the (*φ*, *λ*) imaging plane Δ*λ*_2_ and is the distance from the −*φ* imaging plane.

With the help of the weighting function, the collected data can be weighted, and then the projection data of the constructed plane can be obtained by interpolation, and finally reconstructed by fan beam scanning and then resampling,

(17) $$\begin{array}{c} {\text{c}}_{u}=c_{qpe}+u*\nabla c+\frac{ld}{2*u+1},u=-U,\cdots ,U,\\ \lambda_{0l}=\left(c_{0}-\left|\frac{c_{0}}{\text{handful}}\right|*\text{handful}\right)*\frac{\lambda_{0}}{\left|\lambda_{ol}\right|},\\ q_{0}\lambda =\left(1-\phi \right)*\text{getmile}\left(t,\lambda \right)+\phi *\text{getmile}\left(t+1,\lambda \right),\lambda <\lambda_{0},\phi =\frac{\lambda_{0l}-\lambda }{\text{options}},\\ q\left(\lambda ,\varphi ,u\right)⟵q_{0}\left(\lambda ,\varphi \right)+\overset{c}{\underset{u=1}{\sum }}\left(h_{k}-g_{k}\right). \end{array}$$

In the above algorithm description, the function of this module is to obtain getmile(t, *λ*) the projection data set (t, *λ*) closest to point *c* in the beam projection through linear interpolation *q*_0_(*φ*). Also, *d* is the number of helical turns and LD is the filter length.

RETRACTED

## 3. Design and Implementation Method of CT Imaging Characteristics and Differential Diagnosis of Pulmonary Tuberculosis and Lung Cancer Based on Visual Sensor

### 3.1. Experimental Subjects

#### 3.1.1. Patients with Secondary Pulmonary Tuberculosis

For secondary pulmonary tuberculosis, in order to demonstrate the effect of sputum bacteria on active CT findings, a control group, the active pulmonary tuberculosis group, was established. A group of tuberculosis bacteria also underwent a series of CT examinations in our hospital, and the sputum smears were positive for Acidobacter and Mycobacterium tuberculosis. Therefore, according to this standard, 80 patients with secondary pulmonary tuberculosis with complete clinical data from 2005 to 2010 in our hospital were collected. After the control group is created, the basic conditions of each control group should be compared to check their balance. Secondary pulmonary tuberculosis cases received routine anti-tuberculosis treatment, and multiple spiral CT examinations were performed before treatment, 6 months after treatment, and 12 months after treatment. The specific selection criteria of patients are shown in Table 1.

As can be seen from Table 1, there were 40 cases of secondary pulmonary tuberculosis, 28 males and 12 females, with a male-to-female ratio of 7 : 3.

#### 3.1.2. Lung Cancer Patients

A total of 320 lung cancer cases diagnosed by pathology in Panorama Medical Imaging Diagnosis Center of a city from September 2015 to September 2018 were collected. Clinical data were provided by the hospital follow-up and medical records room. All patients underwent PET/CT scans before surgery or pathological biopsy, and all pathological specimens were tested for ALK. According to clinical criteria, lung cancer is divided into 5 stages, and the number of cases corresponding to each stage is shown in Table 2.

RETRACTED

### 3.2. Inspection Method

For MSCT examination, CT models include P-16 slice helical CT and VCT 16 slice helical CT scan. The specific scanning parameters are shown in Table 3.

With the patient in a supine position, the patient was asked to hold his breath at the end of inspiration and scanned from the patient's thoracic inlet to the bottom of the lung. Multiplanar reconstruction was performed using Simmons and GA 4.0 post-processing workstations to reconstruct coronal and sagittal views if necessary; maximum projected density was also used to visualize vessels around the lesion.

### 3.3. Image Analysis

Two experienced radiologists with the title of deputy director of radiology and above will independently perform the imaging analysis of the nodules without knowledge of the patient's clinical history and pathological findings. If two radiologists have a different diagnosis, they will consult together. The imaging diagnosis opinions were finally agreed, and the location of the nodules (right upper lobe, middle lobe, lower lobe, left upper lobe, lower lobe), diameter, density, and distance from the pleura were recorded. The imaging features of the lesions were then analyzed, including morphology (round or oval, irregular), borders (clear, fuzzy), ear (lobular scars, abrasions, etc.), and internal systems (cavitation marks, cough marks, etc.). Diagnostic criteria are seen in Table 4.

Then, the CT image is input to the main board, and the visual sensor is used for acquisition and processing. The interface board is designed according to two-channel image matching, and each channel has 5-channel signals. The distribution of their connections to the vision sensor main processor board is shown in Table 5.

### 3.4. Pathological Features

In this group of 45 patients with lung disease, 25 were male, 20 were female, 2 had paroxysmal chest pain, and the rest had typical symptoms or needed physical examination. The fluid fractions in the lungs and other nodules were divided into five groups based on cancer results. The consistency analysis results of the diameter and plain CT values of the five groups of cases measured by two observers were all between 0.82 and 0.88, with good consistency.

The chi-square test was used to compare the diameters and CT values of lymph node segments in the five groups of cases: as shown in Figure 7.

As can be seen from Figure 7, there were differences in nodule diameter among the five groups (*F* =16.99, *P* < 0.01). There were extremely significant differences between lung cancer and the other four groups (*P* < 0.01); there were differences in the CT values of nodules in the five groups (*F* =10.01, *P* < 0.01); there were differences in the nodule CT values between the pulmonary tuberculosis group and the lung cancer group, the intrapulmonary lymph node group and the pneumonia group. The difference was statistically significant (*P* < 0.06), and there was no significant difference between the intrapulmonary lymph node group and the pneumonia group, and the lung cancer group and the pneumonia group (*P* > 0.06). The ROC image curve was used to analyze the pulmonary tuberculosis group and the lung cancer group, the accuracy of the CT value of the intrapulmonary lymph node group and the lung hamartoma group, the degree of feature recognition, and the critical value of edge detection (as shown in Figure 8).

RETRACTED

From the ROC curves of the CT values of the pulmonary tuberculosis group and the lung cancer group, it can be seen that the AUC value is 0.788, which is the largest among them, the sensitivity and specificity are 96.5% and 76.1%, respectively, and the diagnostic cutoff value is 27.8Hu. The AUC value was 0.650, the sensitivity and specificity were 90.1% and 74.2%, respectively, and the diagnostic cutoff value was 31.3Hu. The comparison of the nodule position and the distance from the pleura in the five groups of cases is shown in Figure 9. The chi-square test was used for the pairwise comparison:

As can be seen from Figure 9, there were differences in the location of nodules among the five groups of cases (*a* =33.411, *P* = 0.004). The lymph nodes of tuberculosis were 21 mm away from the pleura, and the lymph nodes of lung cancer were 15 mm away from the pleura. There was a statistical difference between the pulmonary tuberculosis group and the lung cancer group.

### 3.5. Algorithm Results

This paper chooses the empty symbol as the mathematical model to explore the effectiveness of the algorithm for analysis and processing.

The cavitation sign refers to the gas density or low-density shadow with a diameter of less than 5 mm in the node, which can be single or multiple. General pathology believes that it generally forms as alveolar spaces that connect with or infiltrate the bronchi, and then the alveoli expand to form cavities. The wall thickness was less than 5, the benign nodules rate was 98%, and the wall thickness was greater than 18 malignant nodules. The segmentation rate is 99%.

The differential diagnosis of a single cavity is based on the size of the lesion, the thickness of the cavity wall, the appearance of the inner and outer edges of the cavity, and the abnormal morphology in and around the cavity.

RETRACTED

The method of judging the cavity sign: First, check whether there is a cavity, count the area of all the cavity, and record it as xo; if it is greater than a given threshold, it means that the lung has a cavity sign.

The hole size and other data are shown in Figure 10.

As can be seen from Figure 10, the number of boundary points in this algorithm can reach more than 140, while the traditional algorithm has only about 100. It can be known that the scope of application of the algorithm in this paper is wider. Furthermore, since vesicle markers and luminal markers share similar morphological features, we can employ a method similar to the chain-code-based multi-region boundary tracking described above to first detect vesicle markers and then analyze them.

## 4. Discuss

The lung is an important gas exchange organ in the human body. It is on the chest. The lungs are divided into lobes, two on the left and three on the right, for a total of five lobes. The Lung Meridian and Lung System (referring to the trachea, bronchi, etc.) are connected with the throat and nose, so the throat is called the portal of the lung, and the nose is the outer orifice of the lung. It can inhale particles, bacteria, viruses, etc. in the air into the alveoli, and has the function of removing foreign bodies. Lung tissue is anatomically divided into parenchymal and interstitial parts. The lung parenchyma includes the bronchi and alveoli at all levels in the lung. The interstitial part of the lung includes connective tissue, blood vessels, and lymphatic vessels and nerves. The interstitium is rich in lymphatic structures (i.e., lymphatic vessels and lymph nodes at all levels in the lungs). The pulmonary lobule is the basic structural and functional unit of lung tissue. There are lobular arteries and bronchioles surrounded by lobular compartments that contain lobular veins, lymphatic vessels, and the interstitium surrounding the pulmonary lobules. The pulmonary lymphatic system plays a pivotal role in the human circulatory system. There are two main functions. One is an important part of the body's defense system and is involved in immune defense; the other is an important aid in the circulatory system, removing mutations and dead cells and eliminating nonself. Foreign bodies maintain the balance of tissue fluid in the body and the stability of the environment.

At present, most researchers believe that low-dose helical CT scan is the first choice for lung disease examination. Reconstruction thickness is up to 0.66 mm. Low-dose helical CT scans have low radiation doses and short scan times. While improving diagnostic accuracy, it also provides increasingly reliable information for patient care. MSCT can perform slice post-reconstruction under low radiation dose scanning conditions, supplemented by multidirectional reconstruction image post-processing technology, to observe lymph node features from multiple angles. It can visualize the three-dimensional shape of lung lesions, accurately locate and diagnose lung lesions, and can clearly show its relationship with surrounding blood vessels, bronchi, and interstitial tissues.

RETRACTED

## 5. In Conclusion

The application of postoperative multidisciplinary spiral CT reconstruction technology reveals tiny and extremely small pulmonary nodules in morphology and three-dimensional morphology, thereby discovering lung cancer and pulmonary tuberculosis that could not be detected and diagnosed in the past and can make accurate diagnosis; to achieve this goal, we use scientific data search method, read data, and adopt and streamline algorithm. Finally, the diagnosis process is optimized. This paper chooses the empty symbol as the mathematical model to explore the effectiveness of the algorithm for analysis and processing. One is to clarify the cavity sign for the appearance of gas density or low-density shadows with a diameter of less than 5 mm in the node, which can be single or multiple. It can be found that the number of boundary points of the algorithm in this paper can reach more than 140, while the traditional algorithm has only about 100. It can be known that the processing range of the algorithm in this paper is wider, and the pathological features can be identified more accurately. The shortcomings of this paper are as follows: First, the current algorithm is only based on the image library collected under laboratory conditions, and the specific application of the algorithm in clinical detection still has a long way to go. Second, the peripheral small cells in this group of studies. There was only 1 case of lung cancer, which could not be evaluated objectively. Further research and evaluation require additional medical records. In the following research and processing, we need to consider the algorithm verification from the images directly collected in the clinic, so that our research cases cover all relevant syndromes of lung diseases and strive to make the research in this paper have broad significance. Through the research of visual sensor, practical suggestions for the study of spiral CT image characteristics are put forward, which has certain theory and significance for the differential diagnosis of secondary pulmonary tuberculosis and the development of lung cancer.

## Figures and Tables

**Figure 1:** Schematic diagram of the CT setup.

RETRACTED

**Figure 2:** Basic structure of helical CT.

**Figure 3:** Projection model.

**Figure 4:** Typical spiral CT image of tuberculosis.

**Figure 5:** Spiral CT image of lung cancer.

**Figure 6:** Structure diagram of general vision sensor.

**Figure 7:** Comparison of nodule diameters and CT values in five groups.

**Figure 8:** ROC curve for CT values.

**Figure 9:** Distance between nodule and pleura in five groups of cases.

**Figure 10:** Invalid symbol analysis data.

**Table 1:** Selection of patients with secondary TB.

Group	Number of cases	Male	Female	Male-to-female ratio	Average age
Secondary pulmonary tuberculosis	40	28	12	7/3	38
Bacterial positive	40	25	15	5/3	44
Bacteria negative	2	1	1	1/1	33

**Table 2:** Selection of lung cancer patients.

	Staging	Number of cases	Average age		Staging	Number of cases	Average age
Observation group	1	48	Twenty-two	Control group	1	33	18
	2	59	26		2	29	Twenty-four
	3	62	25		3	36	Twenty-three
	4	61	31		4	41	Twenty-two
	5	48	37		5	40	26

**Table 3:** Scan parameters.

Parameter	Data	Parameter	Data
Tube voltage	220 V	Mediastinal window	4.5 mm
Tube current	240 mV	Scan layer thickness	4.5 mm
Asphalt	0.912, 1.01	Layer spacing	1.32 mm
Lung window	1360 HV	Image transmission	GA 4.0

**Table 4:** Diagnostic criteria.

Standard	Scope	Standard	Scope
Differences in CT values	22UH	Tumor diameter	>28 mm
Moderate enhancement difference	30UH	Lymph node short diameter	>9 mm
Significant reinforcement difference	>44UH	Lymph node diameter	>13 mm
Nodule diameter	<27 mm	Frozen mediastinum	>28 mm

**Table 5:** Control signal distribution.

Pin	2	4	6	8	10	12	14	16
Signal	Headquarters 3	Headquarters 8	How	Headquarters 10	Headquarters 15	MZZ	How	Headquarters 5
Function	SE110	IN20	0	ERT115	FJ100	1	0	STG110

Pin	18	20	Twenty-two	Twenty-four	26	28	30	32
Signal	E.g	STK	YP1.0	RS2.0	UC3.0	ZE4.0	UPC10.0	HQ 5.0
Function	Sound effect	0	1	FEE1.0	IN1.0	0	FO0.0	ZG1.0

## Data Availability

No data were used to support this study.
